# Application of Big Data Technology and Visual Neural Network in Emotional Expression Analysis of Oil Painting Theme Creation in Public Environment

**DOI:** 10.1155/2022/7364473

**Published:** 2022-09-28

**Authors:** HanZe Guo, XinYu Liang, Yawei Yu

**Affiliations:** School of Fine Arts, Yunnan Normal University, Kunming, Yunnan 650500, China

## Abstract

With the progress of science and technology and the arrival of the big data era, people increasingly rely on computers to deal with daily life and related affairs. In recent years, machine learning has become more and more popular and has achieved good results in some fields, which also makes machine learning widely used. Among them, visual neural network technology can more intelligently analyze the emotional expression of oil painting, which is one of the current research hotspots, involving machine vision, pattern recognition, image processing, artificial intelligence, and other fields. However, in the art field, oil painting is still very different from other images. At present, there is no deep learning algorithm to identify the application of emotional expression analysis in oil painting theme creation. This paper will start with the neural network algorithm and combine the big data recognition technology to analyze the emotional expression of the oil painting subject in the public environment and establish the emotional expression analysis model of oil painting creation based on big data and neural network. The experiment shows that the graphics synthesized by this model have high resolution and good definition, but the speed is slow in the process of experimental operation. It takes about one hour to complete a round of image optimization.

## 1. Introduction

With the rapid economic development of the times, people gradually pursue spiritual culture. In this new era, public art plays a role in improving people's spiritual culture and beautifying the city. As an art culture with a long history, oil painting is not only a way to improve the beautification of urban public environment but also the most effective way to spread culture. Since ancient times, artistic creation has always been a skill that human beings rely on. Excellent paintings reflect human imagination and creativity.

Oil painting originated in Europe in the 15th century and was invented by the Dutch. With the hiding power and transparency of pigments, it can fully express the painted objects, with rich colors and strong three-dimensional texture. For more than 500 years, oil painting has been favored by painters, especially Mona Lisa, the last judgment, Adam and Eve, and other works. Oil painting is a form of painting in which linseed oil, walnut oil, poppy oil, and other quick drying oils, as well as treated Matty resin or Dame resin, are mixed with various color powders to make oil paint and media, and painted on linen, wood, or cardboard. But the algorithm used in the process of painting has always been regarded as a black box model. As for people, painting has always been regarded as a talent. Oil painting requires not only complicated material preparation but also a solid painting foundation. For ordinary people, it is very difficult to complete a professional oil painting. People use computers to convert pictures into different styles. Professional image processing software such as Photoshop can render and adjust the color and curve of photos and render photos into oil painting style, but computers cannot independently create paintings of any style. Recently, the PRISMA laboratory development team from Moscow, Russia, developed a photo editor PRISMA, which combines ordinary photos with the styles of many oil painting artists' works through image stylization and turns them into an oil painting art photo with high perception, beautification, multistyle, etc.

Three scientists from the German Research Canter [1] for integrated neuroscience and theoretical physics published the latest research paper saying that computers can imitate world-famous painters to create oil paintings in 2015. The algorithm proposed by them simulates the processing method of human vision. The first step of creation is to have the feelings you want to express and have a strong desire to act. This is a very important step in the process of creation. How to produce the emotion you want to express? Some situations that we have experienced and felt personally or images that only exist in our minds can make us produce the emotions we want to express. It may be joyful or sad, soft or intense, which will inject emotion and soul into our works [2, 3].

Although the artistic neural network algorithm proposed by German scientists can enable computers to create exquisite works of art, the drawback is that it is a great test for both the computing speed and memory capacity of computers, generating a 512 × 512-pixel painting; in the case of CPU calculation, the calculation time is in hours, which requires at least 16 g of memory. In the case of CPU calculation, the calculation time is in minutes, which requires about 4 GB of video memory. Johnson et al. [4] of Stanford University made improvements to the algorithm, generating pictures and can shift videos style in 2016.

In recent years, machine learning has become more and more popular, especially deep learning has achieved good results in some fields, which also makes deep learning widely used. Deep learning is a branch of machine learning, which combines low-level features to form more abstract high-level features and simulates the mechanism of human brain to interpret data information. Deep learning can achieve good recognition rate in natural scenes, handwriting fonts, face recognition, and Imagenet image database. However, in the art field, there are great differences between artificial oil painting and image graphics in other fields [5]. At present, there is no deep learning algorithm to analyze the emotional expression in oil painting theme creation. Convolutional neural network is a kind of artificial neural network. Due to the use of local convolution and weight sharing, the number of weights can be greatly reduced, thus reducing the complexity of the entire network and improving the operation efficiency. Therefore, convolutional neural network has become a research hotspot of deep learning. Lee and others [6]improved the algorithm by additionally notifying texture transfer with edge direction information. Because only low-level image features at pixel level are used, these algorithms have great limitations in flexibility, effectiveness, diversity, and so on, so the universality of these algorithms is not strong. Despite these methods, and for specific task objectives, a large number of manual parameters are often required.

The historical inevitability of the application of contemporary emotional expression in oil painting creation adapts to and shows the state of personalized development, which is of great significance to the oil painting creation of future artists. At the same time, it also encourages painting creators to pursue their own emotional expression, give full play to their personal style, and respect the diversity of cultural development. This paper discusses the application of big data technology and visual neural network in the emotional expression analysis of oil painting theme creation in the public environment. The innovative application of these two methods realizes the logic part of TensorFlow framework, better determines the skills of creating oil paintings based on emotional expression, and contributes to better artistic creation. It also introduces the application of convolutional neural network in oil painting stylization and shows how to use the characteristics of high-performance convolutional neural network to transfer image styles between images.

## 2. Neural Network and Big Data Technology

### 2.1. Neural Networks and Deep Learning

Hinton published an article that opened the tide of in-depth learning in academia and industry in the 2006 Academic Journal Science. It is a widely parallel connected network composed of adaptive neurons. Its organization can simulate the response of biological neural system to real-world objects [7]. Neural network is the intersection of machine learning and biological science. It is a widely parallel connected network composed of adaptive neurons. Its organization can simulate the response of biological neural system to real world objects. The neuron model has laid the foundation for the development of neural network model.  Figure 1 shows the earliest and simplest “M-P neuron model.”

The weight of M-P network is fixed. For excitatory synapses, the weight is 1; for inhibitory synapses, the weight is -1. In the sequence of signal fault events, when a signal is in the conditional state of 1 to support the occurrence of fault events, the signal connection is excitable; on the contrary, if the state of 1 negates the occurrence of the fault event, the connection is inhibitive. In addition, the input and output of the network are binary variables, and the response function is a step function. Although M-P model is simple, it reflects the main characteristics of biological neurons and can complete any finite logical operations. Common activation functions include sigmoid function, tanh function, and ReLu function. The function diagram of three activation functions is shown in Figure 2.

### 2.2. Convolutional Neural Network

Convolutional neural networks have been studied for nearly 50 years, from the concept of receptive field in biological research in the 1960s to the establishment of the first receptive field-based model in the 1980s. In 1998, the lenet-5 model PW proposed by Lecun of New York University made a breakthrough in handwriting recognition, thus opening the door for convolutional neural network research. In recent years, the holding of the Olympic lmageNet competition in the field of image recognition has pushed the research of convolutional neural networks to a climax. Key universities and laboratories around the world and technology companies have used their trained models for the recognition of ImageNet image library. The champion in 2012 proposed the AlexNet foot model; various networks can be built through CNN, such as cifar10 for natural scenes, LeNet-5 for handwritten fonts as shown in Figure 3, AlexNet for ILSVRC dataset, deep VGG model, etc. These convolutional neural networks aim at different datasets or different objects, and their design network layers and initial design network parameters are different. So far, CNN's design ideas are basically towards deeper networks and more convolution computing [8]. Although the classification accuracy has been improved, it also puts forward higher requirements for the experimental environment. In most depth learning algorithms, the depth of the network is a very important parameter, and the depth convolution neural network is no exception. However, under the condition of relatively small datasets and limited experimental environment, there is no need for a network architecture such as GoogLeNet and deep residual learning, and better results cannot be achieved under such a network architecture. The use of which is briefly introduced below in the part of this article [9].

Convolutional neural network is widely used in image classification, semantic segmentation, feature extraction, style transfer, and so on [10]. For example, a convolutional neural network based on attention mechanism to solve the problem of image classification in complex scenes are proposed. This model is proficient in fine-grained classification and has better robustness [11–13]. The process of convolution is the process of feature extraction. Each convolution kernel represents a feature. If the result of a certain area in the image is larger than that of a convolution kernel, the area is more similar to that convolution kernel. The VGG16 model without full connection layer is selected for image stylization, which includes 13 convolution layers and 5 maximum pooling layers. The performance is improved by continuously deepening the network structure. VGG16 model is divided into five layers. In the first two layers, each layer is pooled after two convolutions, and the last three layers are pooled after three convolutions [14]. Each convolution is accompanied by an activation function. Here, more convolution kernels can make the decision function more discriminative. The overall convolution kernel size is 3 × 3. The effect of three convolution layers in series is not only equivalent to a 7 × 7 convolution layer, which can reduce the parameters of convolution layer, but also has more nonlinear transformations, so that CNN has a stronger ability to learn features. Here, pooling is the maximum pooling, and the size of the pooled core is 2 × 2. Maxpool is easier to capture changes in images and gradients, which brings greater local information differences and better describes the details of edges, textures, and other semantic information. This is especially reflected in network visualization, which visualizes the filter of vgg16 through the gradient rise in the input space. The model is public and can be downloaded in caffe framework [15–18]. The visual structure of each filter is shown in Figure 3. It can be seen that the convolution check color at the lower level has higher edge signal sensitivity, and the higher the convolution core, the more abstract and complex the content is. Image features are extracted by convolution neural network, and different features are extracted by different convolution kernels. A given input image is processed into a group of characteristic images at each processing stage in CNN. The bottom layer mainly reflects the bottom characteristics of pixel level, while the top layer mainly reflects the edge structure of the image [19].

#### 2.2.1. Convolution Layer (Conv Layer)

The traditional neural network adopts the fully connected working mode, which has a poor effect on large-scale digital images. Take a 100∗100∗3 image as an example, each neuron needs to connect 30000 weights, and one layer of network connection will generate millions of weights. Therefore, the fully connected neural network is inefficient and will produce overfitting. Since the concept of receptive field is introduced into the convolutional neural network, in the model, we convert the receptive field into a convolution kernel model, and the convolution kernel parameters are shared. Each layer is composed of a group of convolution kernels, so the weight parameters are greatly reduced. Generally, convolutional neural network model is composed of convolution layer, pooling layer, and full connection layer.

Conv layer is an important part of constructing Conv neural network model [18]. The size of these filters is consistent in space, and the depth of the filter is the same as that of the input data. The VGG network used below is taken as an example. The Conv layer of the first layer of VGG network can be expressed as [64, 3, 3, 3], in which 64, 3, 3, and 3 are called superparameters, which, respectively, represent the number, depth, length, and height of filter banks. In the training process of forward propagation, each group of filters slides up and down, left and right according to the specified step size on the input, then calculates at the sliding box. When the filter slides along the input data, a two-dimensional activation diagram will be generated. The diagram is input on filter and represents a certain feature of the image. For example, the shallow activation diagram is corner information, and the deep activation diagram is an organic combination of shallow layers, representing more complex information.

#### 2.2.2. Pool Layer

At present, most convolutional neural networks have a pool layer embedded in the structure; the purpose of pooling layer is to improve the performance and robustness of the algorithm. It is generally divided into nonoverlapping pooling and overlapping pooling. In this study, the pooling algorithm with overlap and maximum value is used to reduce over fitting. The pooling layer can adopt the maximum value or average value operation. It operates for each depth layer of input data, reducing the size of the data body. Taking VGG network as an example, the pooling layer of VGG network includes two super parameters, namely, space size *F* = 2 and step size *S* = 2. After pooling the input data, 75% of the information is lost, thus avoiding over fitting.

#### 2.2.3. Full Connection Layer

In the fully connected layer of convolutional neural network, neurons are fully connected to all input data in the previous layer, which is the same as that of ordinary neural networks. The full connection layer is mainly used to map the previously learned distribution features into the sample space, thus playing the role of classification. However, due to the parameter redundancy of the full connection layer, some models have adopted other methods to replace the full connection layer to avoid parameter redundancy and have achieved good results.

#### 2.2.4. Optimization Algorithm

In Conv neural networks, the initial parameters of Conv layer filters are randomly generated, and they will produce loss functions in the training process of forward propagation. The parameters of the filter to reduce the loss are optimized in back-propagation. This method of updating the filter parameters by back-propagation is called optimization algorithm. Common optimization methods include random gradient descent method [20], Adam, and L-BFGS. Choosing the appropriate optimization algorithm under specific conditions will have a great impact on the training results of the network. Next, we will briefly introduce Adam and L-BFGS algorithms.

Adam optimization algorithm is an adaptive learning rate optimization algorithm, which was first proposed at the ICLR conference in 2015 [21]. Adam algorithm can be understood as a learning rate adaptive optimizer with momentum method. It is an extension of the random gradient descent method and can replace the classical random gradient descent method to update the network weight more effectively. It estimates the first and second moments of the gradient of each parameter according to the objective function and uses the exponential moving average to calculate. The feature scaling of the gradient of each parameter is unchanged, to solve the problems of high noise and gradient dilution in the process of parameter space iteration.

L-BFGS algorithm [22] is one of the most effective quasi-Newton methods to solve unconstrained optimization problems, with good numerical results and theoretical convergence. This method approximates the Hesse matrix of the objective function by updating the symmetric matrix *Bk*, so that it satisfies the secant equation (quasi-Newton condition). It can be regarded as the conjugate gradient method with additional storage to accelerate the convergence rate, and it can also be regarded as the BFGS method with limited storage. It not only overcomes the difficulty of large amount of calculation of quasi-Newton method but also maintains good convergence. It can be predicted that by modifying the secant equation, we can not only maintain most of the excellent properties of the quasi-Newton method but also better approximate the second-order curvature information of the objective function.

#### 2.2.5. Illustration2Vec

Illustration2vec, that is, the automatic description of illustrations or comics, was first proposed by Saito and Matsui [23] to find matching illustrations for text (as shown in Table 1). They extracted the semantic vector representation of illustrations by training convolutional neural network. The model structure of illustration2vec is similar to that of VGG, but it is a little shallower than the VGG structure introduced above, and it removes all the connection layers and replaces the SoftMax function with sigmoid function. In this paper, the focus is not to discuss how to automatically describe comics. Its model is trained and generated by comics, and its trained model is used for the realization of emotional expression.

#### 2.2.6. VGGNet

The VGG model used in this application is VGG-19 model. The network structure of VGG is easy to understand, because the whole network structure of VGG maintains a very neat structure, and the whole network uses 3× Conv kernel of 3 and 2 × 2. In VGG, the Conv layer is 2 in steps of 1× the Conv of 2 uses the zero padding of 1, which is the same size as the input data volume. The pool layer is 2 with a core of size 2× the maximum value of 2 pooled.  Figure 4 shows the convolutional neural network model.

### 2.3. Big Data Technology

It is a dataset with huge data volume, high data quality, and various data types. Due to these characteristics, it is difficult to rely on traditional tools to capture, process, and manage these big data. Therefore, big data technology should be born. Big data technology integrates several different technical advantages, such as collection, data storage, retrieval, data access, mining, and use; it can realize the rapid processing, analysis, and transmission of huge datasets [24], such as intelligent data screening, analysis, and calculation, to quickly realize the analysis and utilization of huge datasets in a short time by relying on the power of machine intelligence. From the perspective of AI, the emergence of the advantages must be based on huge data. Technology provides important support and assistance for AI [25]. In particular, as the main research direction of knowledge representation, robotics, AI, vision, automatic reasoning, natural language processing, machine learning, etc., although from the perspective of research direction, these contents have their own particularity, and there are certain differences in research methods and main contents. However, all of them need the support of big data technology and need to go through data collation, data collection, algorithm training, algorithm design, and other related processes to achieve the research purpose. Big data technology architecture is shown in Figure 5.

Therefore, the core part of AI is big data technology. The application of big data technology in the field of AI is bound to provide a great auxiliary effect for the development of AI research activities [26]. Especially at the moment of advocating intelligent reform, with the increasing expansion of the application field of AI, the amount of data involved in AI research is gradually increasing, and the research difficulty is increasing. From this point of view, big data technology can exist as an important data processing means of AI. The integration of big data technology and AI can play a good auxiliary and supporting significance [27].

As a technical science, big data mainly studies the simulation of human intelligent activities by machines, so that computers can replace human beings in complex intellectual labor. In the early 1950s, Lebowski successfully used computers to create artificial intelligence artworks, such as waveforms, through repeated research. Harold Cohen developed the art creation software Aaron in 1973 and began to automatically create portraits and still life paintings with certain artistic styles. In addition, through the study of the elements of traditional Chinese ink painting, such as material, media, and artistic effect, as well as the complex relationship elements such as their interaction, the computer drawing system simulating Chinese ink painting has been constructed, and now, it has been able to successfully draw the effect of Chinese painting with ink charm. It is also a general trend that traditional easel oil painting creation is “artificial intelligence.” This impact will affect the creation of easel oil painting as a “pure art” from the aspects of artistic creation, viewing, cultural value, and communication mode. Kurzweil of the United States is even more whimsical: robots will be comparable to human intelligence in 2045. They will acquire “personality” and create works of art “equal” to human intelligence.

## 3. Emotional Expression Analysis Model of Oil Painting Creation Based on Big Data and Neural Network

### 3.1. Feature Style Generation

Convolutional neural networks deal with visual information hierarchically in a feedforward manner. The unit of each layer is the set of image filters. Each image filter extracts a certain feature from the input image and inputs different filters to obtain different feature maps. After the convolution neural network is trained, the object information is more and more clear along the processing level. Along the processing level of the network, the input image pays more and more attention to the actual content of the image and its detailed pixel value. The information about the input image contained in each layer is visualized by reconstructing the image [28] from only the feature map in that layer. The stylization algorithm of convolutional neural network is a texture transmission algorithm, which constrains the texture synthesis method through the feature representation of the most advanced convolutional neural network. A new image is generated by performing a pre image search to match the feature representation of the example image. Therefore, this section will generate the texture feature style of art works from noisy images through Conv neural network, and Figure 6 shows the flow diagram.

The Conv kernel moves 2 horizontally and vertically in the image, so the pooled image is the hit of the input image, and overfitting is avoided. The excitation function of neurons is ReLu function. Relevant research shows that ReLu function has better effect in CNN operation than other traditional function and solves the ingenious problem of explosion. You can directly call the ReLu function in TensorFlow. The correlation degree of different filters can be expressed by Gram matrix *G* of Formula (1), where each element *g*_*ij*_ is the inner product of vectorized characteristic graphs *i* and *j*, as shown in Equation (2). The image is generated step by step through the loss of each layer, which can be expressed by normalization Formula (3). The total loss can be expressed by Equation (4).

(1) $$\begin{array}{c} G=\left[\begin{array}{cccc} g_{11} & g_{12} & \cdots & g_{1n}\\ g_{21} & g_{22} & \cdots & g_{2n}\\ \cdots & \cdots & \cdots & \cdots \\ g_{n1} & g_{n2} & \cdots & g_{nn} \end{array}\right], \end{array}$$

(2) $$\begin{array}{c} g_{ij}=\underset{k}{\sum }F_{ik}F_{jk}, \end{array}$$

(3) $$\begin{array}{c} E=\frac{1}{4N^{2}M^{2}}\underset{i,j}{\sum }{\left(G_{ij}-A_{ij}\right)}^{2}, \end{array}$$

(4) $$\begin{array}{c} L_{\text{style}}=\overset{L}{\underset{l=0}{\sum }}w_{l}E_{l}. \end{array}$$

After completing the theoretical analysis part, you also need to build code in TensorFlow to complete the specific operation process. TensorFlow adopts the operation mode of data flow graph, which is embodied in the fact that the process we become is only to build a data operation process, rather than to implement a specific operation. The specific operation can only be started in one session, and the running process will be completed in the CPU. The result of the operation will be retrieved after the calculation. The advantage of this is to avoid the waste of time and unit width caused by the frequent transmission of data between the CPU video memory and the computer memory [29].

### 3.2. Emotional Expression Analysis

A very important point in oil painting creation is emotion. It has not only become the engine of painting creation but also become a way to vent the author's inner spiritual world. Of course, creators living in different environments have different perceptions. Therefore, the methods, contents, themes, and forms of expression are also quite different. Each art master has formed a unique style by combining his own characteristics [30]. Da Vinci is good at setting off the emotions of characters with the help of composition, which makes his works full of creativity.

Emotion is the most common phenomenon in human life, and it also plays a unique charm in painting. But in today's painting creation, many painters only pay attention to form, thus ignoring the role of emotion. Kandinsky [31] believes that today's art pursues unremitting material and media, and works have gradually become commodities. The phenomenon that emotional and spiritual connotation are ignored in painting does exist; Langer [32] expounds the relationship between emotion and art. Domestic scholars have also made some research achievements. Lingli [33] discussed the influence and importance of emotion on oil painting creation and her understanding and analysis of emotion in oil painting creation. Bi [34] deeply explored the position of emotion in painting creation and said that the process of oil painting creation is the process of painting on the one hand, and the process of expressing the author's inner feelings on the other hand.

The style content of the composite image is different from the other two images that provide content and style, respectively. The image content and the wind cannot be completely separated. Generally, there is no image that completely matches the two constraints at the same time. We will optimize the generated image according to the loss function of the content and style. Each layer in the network defines a nonlinear filter bank, and its complexity increases with the position of the middle layer in the network. In order to analyze the emotional expression in oil painting, this paper also needs the forward propagation of content pictures through Conv neural network model. We can use the functions in the TensorFlow function library to optimize. In order to intuitively show the convergence process of style loss, content loss, noise picture pixel loss, and total loss in the training process, we use tensor board to visualize the decreasing trend of loss and summarize all loss variables through code. At present, the accuracy of emotional evaluation is evaluated from two aspects: first, people's subjective evaluation. Human beings have formed a unique evaluation of artistic beauty in the long-term practice process. The disadvantage of sample delivery is that it cannot form a unified standard. Second, judge the quality of generated pictures through quantitative indicators [35]. Picture loss is a good indicator. Usually, pictures with small loss have relatively evaluation of generated pictures.

## 4. Experimental Test and Analysis

### 4.1. Effect Analysis of Different Styles of Oil Painting

The convolutional neural network used in this algorithm can be well separated from the content and style representations, so the two representations can be processed independently to generate new perceptually meaningful images. The following are the oil painting renderings realized according to the coding. We combine different picture content expression forms with the style expression forms of several oil painting works. In order to ensure the accuracy of emotion analysis and training efficiency, the Conv neural network used in this algorithm can well separate the content and style representation. We combine different image content expression forms with the style expression forms of multiple oil painting works of art.  Figure 7 shows the renderings of different images combined with various oil painting works.

One influencing factor of image stylization is the ratio of *α* and *β*.  Figure 7 shows the content diagram composition of sand painting style, in which *α* and *β* is selected 1 × 10^−2^, 1 × 10^−4^, and 1 × 10^−6^, respectively. From Figure 7, the ratio of *α* and *β* is reduced in turn, that is, the composite image on the left emphasizes the content, which can clearly identify the content, but the style effect of the image is not very good, and the style effect of the image on the right is obvious, but the displayed content is not easy to identify. Color plays a vital role in the rendering of emotion. For example, in the new year, the streets and alleys will be decorated with red decorations; Red Spring Festival couplets will also be pasted on the doors of every household, and a peaceful and lively atmosphere will spontaneously arise. Back to our creation, the same is true.

Figure 8 shows the matching different content feature layer renderings. It can be seen that the essence of artistic creation cannot be separated from “creation.” From experience to conception and then to expression, it is an important stage in the process of artistic creation. Artistic creation is a unique and highly creative spiritual and practical activity of mankind. With the help of various media, through the unique form of artistic language, human beings creatively express their individual survival experience, aesthetic experience, ideas, and so on through artistic images, forming artistic works. It can be seen that every work of art has its unique creative process, and the finiteness and uniqueness of the soul make human art great. The finiteness of life is one of the driving forces of artistic creation and the vitality of artistic works. The unique life experience of artistic creation creates the uniqueness of artistic creation.

### 4.2. Analysis of Emotion Expression in Different Styles of Oil Painting

In order to verify the classification effect of the model, the model is compared with the baseline model selected in this chapter in two classification and three classification experiments on three datasets, and the accuracy of the model is counted. Among them, the second classification experiment classifies the emotional polarity of aspect words into positive and negative, and the third classification experiment classifies the emotional polarity of aspect words into positive, neutral, and negative. In the two classification experiments carried out on three datasets, the accuracy values obtained by different models are shown in Table 2.

It can be seen from Table 2 that the accuracy of this model in three datasets and three different oil painting styles is about 70%, and the values of std. (i.e., standard deviation) are all within a controllable range, which fully shows that the model established in this paper is suitable for emotional analysis tasks of different oil painting styles, because this model can model the forward and backward features of the text at the same time. However, the model does not take into account the emotional features, part of speech features, and the location information between words and aspects in the sentence, so the feature extraction ability is limited. Although the best classification effect is achieved in the baseline model, the model does not introduce emotional features and part of speech features, nor does it consider the impact of location information on the classification results. The model in this paper also needs to consider these factors and further strengthen the analytical ability of the model.

## 5. Discussion and Conclusion

With the advent of the era of big data, oil painting creation needs to keep pace with the times, and it is imperative to create momentum by combining neural network algorithm. Convolutional neural network and big data technology are introduced, and based on these two methods, an emotional expression analysis model of oil painting creation based on big data and neural network is established in this paper. The model is composed of feature style generation and emotion expression analysis, and the effectiveness of this model is verified by experiments. It is found that different styles of oil paintings express different emotions. Although the visual image with high perceptual quality is synthesized, the algorithm still has some technical limitations. The most obvious disadvantage is that the resolution of the synthesized image is low, the definition is greatly reduced, and the speed is slow during the experimental operation. It takes about one hour to complete a round of image optimization. For human society, all innovation must serve people. Whether art or technology, we need to pay attention to and take care of the needs of human beings at the material and spiritual levels, and take this as the bottom line for innovation. AI artistic creation will bring more opportunities for the growth and extension of on-board oil painting creation and exist as a branch of art, which will add more prosperity and splendor to human social life and spiritual world.

## Figures and Tables

**Figure 1:** M-P neuron structure.

**Figure 2:** Function curve.

**Figure 3:** Schematic diagram of LeNet convolution network.

**Figure 4:** Convolutional neural network model.

**Figure 5:** Big data technology architecture.

**Figure 6:** Flow chart of feature style generation.

**Figure 7:** Composition of oil painting styles with different emotional expressions.

**Figure 8:** Matching different content feature layer renderings.

**Table 1:** Illustration2vec structure table.

Input 224 × 224 × 3 RGB image
Conv1_1 + Maxpool
Conv2_1 + Maxpool
Conv3_1 + Conv3_2 + Maxpool
Conv4_1 + Conv4_2 + Maxpool
Conv5_1 + Conv5_2 + Maxpool
Sigmoid

**Table 2:** Comparison of three classification experimental results of the model on three datasets.

Group	Style 1		Style 2		Style 3		Style 4	
	Accuracy	Std.	Accuracy	Std.	Accuracy	Std.	Accuracy	Std.
Dataset 1	0.743	0.159	0.668	0.205	0.678	0.156	0.658	0.098
Dataset 2	0.752	0.063	0.691	0.096	0.682	0.063	0.659	0.069
Dataset 3	0.772	0.136	0.687	0.106	0.701	0.042	0.684	0.123

## Data Availability

The data used to support the findings of this study are available from the corresponding author upon request.
